The article "Efficacy of Self-Made Hewei Decoction for Chronic Atrophic Gastritis and Its Effect on Gastrin and Pepsinogen Expression Levels" was retracted in 2023. Reasons: signs of a paper mill; suspected computer-generated content; unreliable results or conclusions; concerns about the data.

# Efficacy of Self-Made *Hewei* Decoction for Chronic Atrophic Gastritis and Its Effect on Gastrin and Pepsinogen Expression Levels

**DOI:** 10.1155/2022/1092695

**Published:** 2022-06-01

**Authors:** Jianyun Ou, Lin Wang

**Affiliations:** ^1^Department of Traditional Chinese Medicine, Changkou Branch of the First People's Hospital Medical Community of Fuyang District, Hangzhou 311411, Zhejiang Province, China; ^2^Department of Integrated Traditional Chinese and Western Medicine, First People's Hospital of Fuyang District, Hangzhou 311400, Zhejiang Province, China

## Abstract

We aim to investigate the therapeutic effect of self-made *Hewei* decoction based on the differences-in-differences (DID) model for treating chronic atrophic gastritis and its effect on the gastrin and pepsinogen expression. A total of 166 chronic atrophic gastritis patients treated in our hospital from January 2019 to September 2020 were recruited and randomly assigned to a treatment group and a control group (*n* = 83 per group). In the control group, patients were given conventional western medicine. In the treatment group, patients were administered self-made *Hewei* decoction besides conventional western medicine. The general data, total effective rate, and histological changes before and after treatment were compared between the two groups. The DID model was utilized to compare the changes in three items of gastric function and traditional Chinese medicine (TCM) syndrome scores at various time points (before treatment and 1, 3, 6, and 12 months after treatment) between the two groups. In the treatment group, 5 cases were lost to follow-up, and 78 cases remained. In the control group, 4 cases were lost to follow-up, and 79 cases remained. The total effective rate in the treatment group (93.59%) was significantly higher than that in the control group (82.28%) (*P* < 0.05). The histological score was not significantly different between the two groups before treatment (*P* > 0.05). The histological score at 12 months after treatment was lower than those before treatment in the two groups (*P* < 0.05). The histological score was lower in the treatment group than that in the control group (*P* < 0.05). After treatment, the TCM syndrome score and PGR17 level were lower in the treatment group than those in the control group at each time point (*P* < 0.05). PGI and PGII levels were higher in the treatment group than those in the control group at each time point (*P* < 0.05). DID regression model showed that TCM syndrome score and PGR17 level decreased by 106.2% and 65.8%, respectively, after treatment in patients with chronic atrophic gastritis (*P* < 0.05), but the treatment mode was opposite to the overall therapeutic effect in terms of time. The PGI and PGII levels increased by 102.9% and 97.8%, respectively, in patients with chronic atrophic gastritis (*P* < 0.05), and the treatment mode was the same as the overall therapeutic effect in terms of time. There was no significant difference in the therapeutic effect between the two groups at 1 month after treatment. A significant difference in the therapeutic effect was detected between the two groups at 3 months after treatment, and the difference showed a decreasing trend after 6 months after treatment. Self-made *Hewei* decoction can improve the histological alterations in chronic atrophic gastritis, relieve clinical symptoms, and ameliorate the expression levels of three items of gastric function.

The article "Efficacy of Self-Made Hewei Decoction for Chronic Atrophic Gastritis and Its Effect on Gastrin and Pepsinogen Expression Levels" was retracted in 2023. Reasons: signs of a paper mill; suspected computer-generated content; unreliable results or conclusions; concerns about the data.

## 1. Introduction

Chronic atrophic gastritis (CAG) is a frequent digestive tract disease and a type of chronic gastritis. CAG is characterized by atrophy of the gastric body and fundus and autoantibodies against parietal cells (PCA) and their secreted intrinsic factors (IFA) in circulation. People affected by other autoimmune diseases have a significantly higher prevalence, often accompanied by pernicious anemia (PA). As a result, CAG is found in 10–15% of children and 15–25% of adults with type 1 diabetes (DM1). The prevalence rate in the general population is 2%, while in DM1 patients, the prevalence rates of the AAG and PA are 5–10% and 2.6–4%, respectively. Up to 1/3 patients with autoimmune thyroid disease (AITD) also detected CAG [1]. The essential pathological features are the reduction in the volume and number of intrinsic glands in the gastric mucosal epithelium and presence or absence of intestinal metaplasia (IM) or atypical hyperplasia (ATP) [2]. The precise pathogenesis remains unclear. It is generally believed to be associated with *Helicobacter pylori* infection, immune factors, and bile reflux. The prolonged duration of the disease and recurrent attack bring huge adverse effects on patients' production and life.

In the category of traditional Chinese medicine (TCM), CAG belongs to “chest-abdominal distension,” “abdominal pain,” and “gastric stuffiness.” Its occurrence is mainly associated with improper diet, emotional disorders, internal invasion of evil and toxin, and inherent deficiency. The treatment needs to strengthen the spleen and stomach [3]. With the development of medicine in China, Chinese medicine has displayed more and more obvious advantages in the treatment of CAG. *Baohe* Pill, *Xiangsha Liujunzi* Decoction, *Banxia Xiexin* Decoction, and *Guipi* Pill have achieved good outcomes for treating CAG [4]. Wu et al. [5] have found that acupuncture combined with *Jiawei Xiangsha Liujunzi* Decoction can remarkably improve gland atrophy and dysplasia and relieve clinical symptoms in CAG patients. In the experiment of Pan and Huang [6], *Jiawei Banxia Xiexin* Decoction can dramatically diminish TCM syndrome score and improve the therapeutic effect. All the above studies have demonstrated that the Chinese medicine formula has obvious effects on the treatment of CAG. The *Hewei* decoction is self-made based on the basic theory of TCM and the combination with the modern pharmacology of TCM. It has certain unique features in the treatment of CAG and has achieved some clinical effects. Nevertheless, data are not sufficient to support the precise improvement and action mechanism. Differences-in-differences (DID) is a data model that can assess policy effects, reduce the interference of endogenous factors, and better evaluate clinical effects. Taken together, this study was designed to observe the clinical effect of the self-made *Hewei* decoction in the treatment of CAG, discuss the TCM syndrome score and gastric function before and after treatment, and analyze the effect of self-made *Hewei* decoction on the histology of CAG patients based on the DID model.

The article "Efficacy of Self-Made Hewei Decoction for Chronic Atrophic Gastritis and Its Effect on Gastrin and Pepsinogen Expression Levels" was retracted in 2023. Reasons: signs of a paper mill; suspected computer-generated content; unreliable results or conclusions; concerns about the data.

## 2. Data and Methods

### 2.1. General Data

The study was approved by the institutional review board of the Chang Kou branch of the First People's Hospital, and the patients and their family members all gave written informed consent. A total of 166 CAG patients diagnosed and treated in our hospital from January 2019 to September 2020 were enrolled as subjects. This study was approved by the hospital ethics committee. Patients and their families signed informed consent. Inclusion criteria were the following: (1) all meeting the diagnostic criteria of western medicine for CAG formulated in the *Chinese Consensus Opinions on Chronic Gastritis* [7] and having undergone gastroscopic biopsy within 1 month; (2) in line with the TCM diagnostic criteria for CAG formulated by the *Guidelines for Clinical Research on New Chinese Medicines* [8], i.e., Syndrome of Deficiency of Spleen *Qi* and Stomach *Qi*, including epigastric pain, persistent pain in the stomach, pain relief after eating, fullness after eating, belching, poor appetite, mental fatigue, yellow and white complexion, fat and pale tongue, thin white or greasy fur, and thin pulse; (3) age between 18 and 80 years, with complete clinical data, ability to cooperate with the whole treatment and examination. Exclusion criteria were the following: (1) patients with malignant tumors of the digestive tract or other malignant tumors; (2) patients with severe gastric or duodenal ulcers; (3) patients with severe liver and kidney insufficiency or rheumatism; (4) a history of severe drug allergies or allergic to medication; (5) mental disorder and inability to cooperate. All subjects were randomly divided into a treatment group (*n* = 83) and a control group (*n* = 83). There were no significant differences in general data such as age and sex between the two groups (*P* > 0.05), as shown in Table 1.

The article "Efficacy of Self-Made Hewei Decoction for Chronic Atrophic Gastritis and Its Effect on Gastrin and Pepsinogen Expression Levels" was retracted in 2023. Reasons: signs of a paper mill; suspected computer-generated content; unreliable results or conclusions; concerns about the data.

### 2.2. Methods

#### 2.2.1. General Information Collection

After enrollment, the patients in the two groups were asked in detail concerning their current illness history, past history, and family history. The basic vital signs such as blood pressure and heart rate were monitored, and the patients were asked about their work and life pressure, work, and rest habits. Tissue biopsy was conducted using gastroscopy. Histological scoring was performed. TCM syndrome score was given. The fasting venous blood was drawn in the morning of the second day to detect three items of gastric function.

#### 2.2.2. Treatment Methods

The control group received dietary adjustment and conventional western medicine treatment. The conventional western medicine treatment was carried out according to the *Chinese Consensus Opinions on Chronic Gastritis* [7] and was given lansoprazole and bismuth potassium citrate capsules. The patients combined with *Helicobacter pylori* infection were additionally treated with amoxicillin and clarithromycin quadruple for treating *Helicobacter pylori* infection for 14 days. Besides the treatment in the control group, patients in the treatment group were subjected to self-made *Hewei* decoction. The prescription contains Bulbus Lilii 30 g, Poria Cocos 30 g, Atractylodes Macrocephala 30 g, Scrophularia Ningpoensis 25 g, Radix Linderae 15 g, Alisma Orientale 30 g, Ophiopogon Japonicus 30 g, Angelica Sinensis 15 g, Corydalis 15 g, Radix Paeoniae Alba 15 g, Caulis Dendrobii 20 g, Anemone Altaica 9 g, Ligusticum Wallichii 9 g, Endothelium Corneum Gigeriae Galli 12 g, Panax notoginseng 6 g, Radix Sanguisorbae 9 g, Pollen Typhae 9 g, and roasted licorice 3 g. One dose was taken daily and the decoction was decocted with water. The decoction was boiled 200 mL each time. After boiling twice, the two decoctions were mixed. The mixture was taken orally in the morning and evening, separately. Both groups were treated for 3 months.

### 2.3. Observation Indicators

#### 2.3.1. Total Effective Rate

(1) Clinical recovery: clinical symptoms and signs disappeared completely (or disappeared), and tissue biopsy improved remarkably; (2) markedly effective: clinical symptoms and signs disappeared significantly, tissue biopsy improved; (3) effective: the clinical symptoms and signs were slightly improved, and the tissue biopsy was slightly improved; (4) ineffective: there is no improvement (or even aggravation) in clinical symptoms and signs and no improvement (or even aggravation) in histology. Total effective rate = (recovery + markedly effective + effective)/total number of cases × 100% [9].

The article "Efficacy of Self-Made Hewei Decoction for Chronic Atrophic Gastritis and Its Effect on Gastrin and Pepsinogen Expression Levels" was retracted in 2023. Reasons: signs of a paper mill; suspected computer-generated content; unreliable results or conclusions; concerns about the data.

#### 2.3.2. TCM Syndrome Score

In accordance with the *Guidelines for Clinical Research on New Chinese Medicines* [8], a TCM syndrome quantitative score table was developed, including epigastric pain, fullness after eating, mental fatigue, thin white or greasy fur, and thin pulse. The symptom was quantitatively scored as 0–3 points according to the degree of symptoms, with a total score of 15. The higher the score, the more severe the symptom. The symptom was scored by two TCM physicians with a fixed intermediate title and a master's degree or above before treatment and 1, 3, 6, and 12 months after treatment.

#### 2.3.3. Histological Score

According to the alteration in a tissue biopsy, a scoring table was developed, containing gland atrophy, intestinal metaplasia, and atypical hyperplasia. According to the degree of change, the symptom was quantitatively scored as 0–3 points, with a total score of 9. The high score indicated severe symptoms. Blind design was used to reduce research bias, and patient symptom information was blindly and randomly graded by two pathologists and workers with a master's degree or above before and after treatment. After that, the two scores were averaged.

#### 2.3.4. Three Items of Gastric Function

Gastrin 17 (PGR17), pepsinogen I (PGI), and pepsinogen II (PGII) were measured before treatment and 1, 3, 6, and 12 months after treatment. 2-3 ml of venous blood was taken from the patient after 8 hours of fasting in the morning on day 2 after enrollment. After centrifugation, the upper serum was obtained to examine the three items of gastric function in Hangzhou ADICON Medical Laboratory Center using a gastric function detector (model: Mokosensor-A300; MOKOBIO Medical Instrument Co., Ltd.).

### 2.4. Follow-Up

A special person was assigned to follow up all patients in the outpatient clinic, once a week in the first three months. The medication was adjusted according to the patient's symptoms. Afterward, the patients were followed up in the outpatient clinic once a month. The changes in the patient's condition were recorded. The patients were instructed to regularly recheck relevant examinations in the outpatient clinic and carry out various scores.

### 2.5. Quality Control

The protocols were reviewed and revised in strict accordance with the inclusion and exclusion criteria. All relevant researchers should be trained to ensure the accuracy and integrity of clinical data. All data were recorded by two persons with double input. Quality control was strictly conducted at each stage of data processing to ensure data accuracy.

The article "Efficacy of Self-Made Hewei Decoction for Chronic Atrophic Gastritis and Its Effect on Gastrin and Pepsinogen Expression Levels" was retracted in 2023. Reasons: signs of a paper mill; suspected computer-generated content; unreliable results or conclusions; concerns about the data.

### 2.6. Statistical Processing

All data were input by Epidata 3.1 and analyzed by Stata 15.0 software. The measurement data that met the normal distribution were expressed as $\left(\bar{\chi }\pm s\right)$. The paired-sample *t*-test was employed for intragroup comparison, and the independent-sample *t*-test was utilized for intergroup comparison. Count data were expressed as a number of cases/constituent ratio *n* (%), and *χ*^2^ test was used. Ranked data were analyzed using rank-sum test. DID method was applied to assess the three items of gastric function in CAG patients after treatment. Dummy variables Treat and Time were set, where Treat = 1 represents the patients in the treatment group; Treat = 0 represents the patients in the control group; Time = 0 represents before treatment; Time = 1, 2, 3, and 4 represent 1, 3, 6, and 12 months after treatment. The DID model could be set as *y* = *β*_0_ + *β*_1_Treat_it_ + *β*_2_Time_it_ + *β*_3_Treat_it_ × Time_it_ + *ε*_it_. The subscripts *i* and *t* represent the group and time, respectively; *ε* is the random disturbance term; Y represents the three items of gastric function. A parallel trend test plot was drawn using the Coefplot package in Stata software. A value of *P* < 0.05 was considered statistically significant.

## 3. Results

### 3.1. Follow-Up Situation

In the treatment group, 5 cases were lost to follow-up, and 78 cases remained. In the control group, 4 cases were lost to follow-up, and 79 cases remained.

### 3.2. Comparison of the Total Effective Rate between the Two Groups

The total effective rate of the treatment group (93.59%) was significantly higher than that of the control group (82.28%) (*P* < 0.05), as shown in Table 2.

### 3.3. Comparison of Histological Scores between the Two Groups before and after Treatment

No significant difference in the histological scores was determined between the two groups before treatment (*P* > 0.05). The histological scores at 12 months after treatment were lower than those before treatment in the two groups (*P* < 0.05), and the score was lower in the treatment group than that in the control group (*P* < 0.05), as shown in Table 3.

### 3.4. Comparison of TCM Syndrome Score at Various Time Points in the Two Groups before and after Treatment

TCM syndrome score was lower in the treatment group than that in the control group at each time point after treatment (*P* < 0.05), as shown in Table 4.

### 3.5. Comparisons of Three Items of Gastric Function in the Two Groups at Various Time Points before and after Treatment

PGI and PGII levels were higher in the treatment group than those in the control group at each time point after treatment (*P* < 0.05). PGR17 level was lower in the treatment group than that in the control group at each time point after treatment (*P* < 0.05), as shown in Table 5.

The article "Efficacy of Self-Made Hewei Decoction for Chronic Atrophic Gastritis and Its Effect on Gastrin and Pepsinogen Expression Levels" was retracted in 2023. Reasons: signs of a paper mill; suspected computer-generated content; unreliable results or conclusions; concerns about the data.

### 3.6. Effects of Different Treatments on TCM Syndrome Score and Three Items of Gastric Function Analyzed Using the DID Model

DID regression model showed that TCM syndrome score and PGR17 level decreased by 106.2% and 65.8% in CAG patients after treatment, respectively (*P* < 0.05), but the treatment mode was opposite to the overall therapeutic effect in terms of time. With the prolonged time, TCM syndrome score and PGR17 level increased by 121.7% and 72.5%, respectively (*P* < 0.05). The PGI and PGII levels increased by 102.9% and 97.8% in CAG patients, respectively (*P* < 0.05), and the treatment mode was the same as the overall therapeutic effect in terms of time. With the prolonged time, PGI and PGII levels increased by 110.5% and 99.3%, respectively (*P* < 0.05), as shown in Table 6.

### 3.7. Effects of Self-Made *Hewei* Decoction on TCM Syndrome Score and Gastric Function in CAG Patients Analyzed by Parallel Trend Test

The parallel trend test was conducted with pretreatment as the baseline period. The results did not exhibit significant differences in the therapeutic effect between the two groups at 1 month after treatment, suggesting that the two groups met the parallel trend assumption before treatment. A significant difference in the therapeutic effect was detected between the two groups at 3 months after treatment, and the difference displayed a decreasing trend 6 months after treatment, as shown in Figures 1to 4.

## 4. Discussion

CAG, a chronic inflammatory disease in the gastric mucosa, has a high incidence and is strongly associated with the occurrence of gastric cancer. It is clinically believed that the disease is associated with *Helicobacter pylori* infection, genetics, and dietary habits [10]. Currently, the conventional methods of western medicine mainly focus on symptomatic treatment and eradication of *Helicobacter pylori* infection, but the clinical effect is not ideal [11]. With people's attention to traditional Chinese medicine, the research addressing the treatment of CAG with integrated traditional Chinese and Western medicine has gradually developed and achieved good results. This disease belongs to “chest-abdominal distension,” “abdominal pain,” and “gastric stuffiness” in the category of traditional Chinese medicine. Weakness of the spleen and stomach is the basic pathogenesis of the CAG. The spleen and stomach are the sources of generating *Qi* and blood and also the hub of the rise and fall of *Qi*. Therefore, when the spleen and stomach are weak, the *Qi* and blood of the human body can be affected. Moreover, improper diet, congenital insufficiency, overwork, emotional internal injury, and exogenous climatic pathogens lead to the stomach failing to send downwards and *Qi* obstruction, which unbalances the body fluid and yang *Qi* in the stomach and induces the occurrence of CAG. Therefore, *Qi* stagnation is important pathogenesis of CAG. The treatment should strengthen the spleen and stomach to activate blood and regulate *Qi*. In the study of Liu et al. [12], *Jiawei Xiaoyao* Powder, which can smooth the liver, regulate *Qi*, and strengthen the spleen and the stomach, has achieved good results in the treatment of CAG with liver depression and spleen deficiency. Wang et al. [13] applied self-made *Tiaowei* decoction to treat CAG and found that MTL and SS were remarkably improved, and the TCM syndromes were relieved. Nevertheless, the current studies regarding the treatment of CAG with integrated traditional Chinese and western medicine mainly focus on the clinical efficacy and risk factors, not the action pathway of the medicine. Furthermore, subjective evaluation indicators such as TCM syndrome score are selected. It is easy to omit some variables, making the results biased.

The article "Efficacy of Self-Made Hewei Decoction for Chronic Atrophic Gastritis and Its Effect on Gastrin and Pepsinogen Expression Levels" was retracted in 2023. Reasons: signs of a paper mill; suspected computer-generated content; unreliable results or conclusions; concerns about the data.

CAG is characterized by the atrophy of the gastric mucosal epithelium and glands. The decreased cell number and volume induce the insufficient secretion of various digestive juices, thereby resulting in abnormal gastric function and abnormal secretion of hormones such as PGI, PGII, and PGR17. The patient presented indigestion, abdominal distension, abdominal pain, loss of appetite, and fatigue. The results from this study demonstrated that the total effective rate of the treatment group was higher than that of the control group. It is indicated that the combination with self-made *Hewei* decoction has better effects on CAG. The self-made *Hewei* decoction is composed of 19 Chinese medicines: Bulbus Lilii, Poria Cocos, Atractylodes Macrocephala, Scrophularia Ningpoensis, Radix Linderae, Alisma Orientale, Ophiopogon Japonicus, Angelica Sinensis, Corydalis, Radix Paeoniae Alba, Caulis Dendrobii, Anemone Altaica, Ligusticum Wallichii, Endothelium Corneum Gigeriae Galli, Panax notoginseng, Radix Sanguisorbae, Pollen Typhae, and roasted licorice. Among them, Bulbus Lilii and Atractylodes Macrocephala are the monarch drugs, which can nourish *Yin* and regulate *Qi*. Nowadays, pharmacology has proven that Bulbus Lilii can promote gastric juice secretion, regulate gastrointestinal nerves, and improve gastric motility [14]. Atractylodes Macrocephala can enhance the spontaneous contraction of the gastrointestinal tract, increase the contraction amplitude, and suppress stress ulcers [15]. The ministerial drugs consist of Panax notoginseng, Endothelium Corneum Gigeriae Galli, Alisma Orientale, Radix Sanguisorbae, Ligusticum Wallichii, and Angelica Sinensis. Panax notoginseng can activate blood and stop bleeding. Ligusticum Wallichii can promote blood circulation, remove blood stasis, and clear collaterals. Radix Sanguisorbae can cool blood and stop bleeding. Angelica Sinensis can nourish the blood. The combined action of the four herbs can anticoagulate, prevent gastric mucosal bleeding, clear the collaterals, remove rot, improve gastric mucosal blood supply and gastric mucosal function, and diminish gastric mucosal damage. Endothelium Corneum Gigeriae Galli, Alisma Orientale, and Angelica Sinensis can invigorate the spleen, remove dampness, and promote digestion. Adjuvant drug Anemone Altaica can clear away heat and dampness. The guiding drugs Radix Paeoniae Alba, Corydalis, Radix Linderae, and roasted licorice can move *Qi*, relieve pain, and regulate *Qi* movement. Modern pharmacological studies have confirmed [16] that Radix Paeoniae Alba can nourish blood and astringe *Yin*, soften the liver, and relieve pain. The combination of Radix Paeoniae Alba and Angelica Sinensis is good for treating liver and spleen disharmony. The combination of Caulis Dendrobii and Ophiopogon Japonicus can reinforce the stomach and regenerate fluid. The combination of Poria Cocos and Atractylodes Macrocephala can strengthen the spleen and dampness and can improve the immune function of the body. The abovementioned herbs together can invigorate the spleen, regulate *Qi*, promote blood circulation and relieve pain, and obviously relieve CAG such as stomach pain, upper abdominal fullness, anorexia, heartburn, and fatigue. The results showed that the histological score and TCM syndrome score of the treatment group were significantly reduced, and the scores were lower than those after western medicine treatment. The self-made *Hewei* decoction has a remarkable effect on the treatment of CAG.

The article "Efficacy of Self-Made Hewei Decoction for Chronic Atrophic Gastritis and Its Effect on Gastrin and Pepsinogen Expression Levels" was retracted in 2023. Reasons: signs of a paper mill; suspected computer-generated content; unreliable results or conclusions; concerns about the data.

From the perspective of modern anatomy, the meridians in the body are significantly associated with small and medium blood vessels and nerves. Various inflammatory cascade reactions caused by them can stimulate the gastrointestinal tract and affect gastric function. The three items of gastric function are important indicators of gastric function. In atrophic gastritis patients, PGI and PGII levels are increased, but PGR17 level is decreased [17]. The more obvious the abnormality, the worse the gastric function of the patient [18]. In the self-made *Hewei* decoction, the monarch drug Bulbus Lilii can regulate the changes in phosphorylated extracellular signal-regulated kinase (p-ERK) and extracellular regulated protein kinase (ERK) expression, improve gastric function, and promote the secretion of various gastric juices [19]. However, Endothelium Corneum Gigeriae Galli and Radix Paeoniae Alba can improve the atrophy of the glands on the gastric mucosa and promote the synthesis and secretion of motilin, gastrin, and pepsinogen I. The combined action of the above-described drugs improves the gastric function of CAG and dramatically reduces the TCM syndrome score. In this study, TCM syndrome score and PGR17 level were lower, while PGI and PGII levels were higher in the treatment group than those in the control group at each time point after treatment. It is indicated that the three items of gastric function and TCM syndromes were significantly improved in the patients treated with the self-made *Hewei* decoction. These findings may be because Bulbus Lilii, Atractylodes Macrocephala, and Endothelium Corneum Gigeriae Galli can increase the synthesis of pepsin by promoting the activation of p-ERK and ERK pathways, promote the secretion of chief cells of the gastric fundus, and can also improve the nutritional status of the gastrointestinal tract by regulating the nerves and microcirculation of the gastrointestinal tract, slow the atrophy of the glandular cells in the stomach, and help to improve the secretion of pepsin. Clinically, when evaluating the treatment of various diseases with TCM, the selection of subjective TCM syndrome score can lead to endogenous factors, which can induce result deviations. As an emerging data model, DID can alleviate the problem of omitted variable bias to a certain extent, reduce the bias caused by dummy variables such as subjective evaluation, and improve the credibility of the results. Thus, the DID model was selected in our hospital to assess the treatment of CAG with self-made *Hewei* decoction, and the DID model was used to compare TCM syndrome score and the three items of gastric function at various time points before and after treatment. Our results exhibited significant differences in therapeutic effect between the two groups, further indicating that the self-made *Hewei* decoction exerts an obvious effect on improving the gastric function of CAG patients. The self-made *Hewei* decoction has a high clinical application value in the treatment of CAG.

## 5. Conclusion

In summary, the self-made *Hewei* decoction can improve the histological changes of CAG patients, alleviate the clinical symptoms, and improve the expression levels of three items of gastric function. However, this study has some limitations, such as a small sample size, resulting in a small amount of statistical data and biased results to a certain extent. This study only observed the improvement of gastric function and TCM syndrome score 12 months after treatment, which has preliminary verified that this decoction plays a certain role in improving gastric function, but the study on the long-term effect is insufficient. Therefore, further investigations with large samples over a long period are required.

The article "Efficacy of Self-Made Hewei Decoction for Chronic Atrophic Gastritis and Its Effect on Gastrin and Pepsinogen Expression Levels" was retracted in 2023. Reasons: signs of a paper mill; suspected computer-generated content; unreliable results or conclusions; concerns about the data.

## Figures and Tables

**Figure 1:** Parallel trend test of self-made *Hewei* decoction effect on TCM syndrome score in patients with chronic atrophic gastritis.

**Figure 2:** Parallel trend test of self-made *Hewei* decoction effect on PGR171 level in patients with chronic atrophic gastritis.

**Figure 3:** Parallel trend test of self-made *Hewei* decoction effect on PGI in patients with chronic atrophic gastritis.

**Figure 4:** Parallel trend test of self-made *Hewei* decoction effect on PGII in patients with chronic atrophic gastritis.

**Table 1:** Comparison of general data between the two groups [*n* (%), $\left(\bar{\chi }\pm s\right)$].

Item		Treatment group (*n* = 83)	Control group (*n* = 83)	*t*/*χ*^2^	*P*
Sex (*n*)	Male	38 (45.78)	35 (42.17)	0.220	0.639
	Female	45 (54.22)	48 (57.83)		
Age (year)		47.70 ± 9.38	46.14 ± 10.09	1.032	0.304
Duration (year)		8.16 ± 2.29	7.85 ± 1.91	0.947	0.345
Family history of chronic atrophic gastritis (*n*)		8 (9.64)	7 (8.43)	0.073	0.787
History of drinking (*n*)		41 (49.40)	39 (46.99)	0.621	0.431
History of smoking (*n*)		19 (22.89)	18 (21.69)	0.097	0.756

Life and work pressure (*n*)	High	55 (66.27)	53 (63.86)	0.106	0.745
	Low	28 (33.73)	30 (36.14)		

Lifestyle (*n*)	Regular work and rest	61 (73.49)	57 (68.67)	0.469	0.493
	Irregular work and rest	22 (26.51)	26 (31.33)		

*Helicobacter pylori* infection	Yes	49 (59.04)	51 (61.45)	0.101	0.751
	No	34 (40.96)	32 (38.55)		

Degree of atrophy	+	39 (46.99)	38 (45.78)	0.296	0.862
	++	27 (32.53)	30 (36.15)		
	+++	17 (20.48)	15 (18.07)		

IM degree	0	28 (33.74)	30 (36.15)	0.241	0.971
	+	23 (27.71)	24 (28.91)		
	++	19 (22.89)	17 (20.48)		
	+++	13 (15.66)	12 (14.46)		

ATP degree	0	35 (42.17)	36 (43.37)	0.111	0.946
	+	29 (34.94)	27 (32.53)		
	++	19 (22.89)	20 (24.10)		

**Table 2:** Comparison of the total effective rate between the treatment and control groups.

Group	Clinical recovery	Markedly effective	Effective	Ineffective	Total effective rate
Treatment (*n* = 78)	18 (23.08)	32 (41.02)	23 (29.49)	5 (6.41)	73 (93.59)
Control (*n* = 79)	12 (15.19)	28 (35.44)	25 (32.05)	14 (17.72)	65 (82.28)
*χ* ^2^					4.721
*P*					0.030

The article "Efficacy of Self-Made Hewei Decoction for Chronic Atrophic Gastritis and Its Effect on Gastrin and Pepsinogen Expression Levels" was retracted in 2023. Reasons: signs of a paper mill; suspected computer-generated content; unreliable results or conclusions; concerns about the data.

**Table 3:** Comparison of histological scores between the treatment and control groups before and after treatment ($\bar{\chi }\pm s$, points).

Group	Before treatment	12 months after treatment	*t*	*P*
Treatment (*n* = 78)	7.12 ± 1.69	4.31 ± 0.73	13.481	<0.001
Control group (*n* = 79)	7.05 ± 1.71	5.58 ± 1.03	6.504	<0.001
*T*	0.258	8.903		
*P*	0.797	<0.001		

**Table 4:** Comparison of TCM syndrome score at different time points before and after treatment in the treatment and control groups $\left(\bar{\chi }\pm s\right)$.

Group	Before treatment	1 month after treatment	3 months after treatment	6 months after treatment	12 months after treatment	*F*	*P*
Treatment (*n* = 78)	13.12 ± 1.72	10.25 ± 1.45	7.23 ± 1.07	6.95 ± 0.95	6.36 ± 0.91	Interaction = 25.757	0.030
Control (*n* = 79)	12.94 ± 1.68	11.11 ± 1.59	9.70 ± 1.41	8.79 ± 1.37	8.67 ± 1.28	Time = 449.521	<0.001
*T*	0.665	3.540	12.353	9.767	13.018	Inter-group = 222.059	0.015
*P*	0.507	0.001	<0.001	<0.001	<0.001		

**Table 5:** Comparison of three items of gastric function at different time points before and after treatment in the treatment and control groups ($\bar{\chi }\pm s$, *n* = 68).

Three items of gastric function	Group	Before treatment	1 month after treatment	3 months after treatment	6 months after treatment	12 months after treatment	*F*	*P*
PGR17 (pg/ml)	Treatment (*n* = 78)	143.74 ± 15.29	123.00 ± 12.48	90.23 ± 9.37	88.95 ± 8.75	86.67 ± 8.61	Interaction = 9.409	0.030
	Control (*n* = 79)	144.01 ± 14.87	134.98 ± 13.20	103.70 ± 10.40	101.64 ± 9.96	99.89 ± 10.03	Time = 157.521	<0.001
	*T*	0.112	5.842	8.523	8.477	8.856	Intergroup = 636.059	0.015
	*P*	0.911	<0.001	<0.001	<0.001	<0.001		

PGI (ng/ml)	Treatment (*n* = 78)	38.86 ± 6.97	50.05 ± 7.82	75.37 ± 9.20	77.68 ± 9.41	78.84 ± 10.04	Interaction = 13.693	<0.001
	Control (*n* = 79)	38.90 ± 6.45	46.67 ± 7.19	65.66 ± 8.41	67.26 ± 8.73	68.04 ± 9.19	Time = 130.110	<0.001
	*T*	0.037	2.820	6.904	7.194	7.032	Intergroup = 568.335	<0.001
	*P*	0.970	0.005	<0.001	<0.001	<0.001		

PGII (ng/ml)	Treatment (*n* = 78)	40.98 ± 6.69	51.43 ± 7.35	77.82 ± 8.38	79.75 ± 8.67	81.05 ± 8.72	Interaction = 24.693	<0.001
	Control (*n* = 79)	41.03 ± 6.88	47.28 ± 6.94	64.47 ± 7.82	66.28 ± 7.93	69.02 ± 7.95	Time = 240.335	<0.001
	*T*	0.046	3.638	10.322	10.160	9.035	Intergroup = 635.312	<0.001
	*P*	0.963	<0.001	<0.001	<0.001	<0.001		

**Table 6:** DID analysis of the effects of different treatments on TCM syndrome score and gastric function.

Index	Variable	Coefficient	Standard error	*t*	*P*	95% *CI*	*P*
TCM syndrome score	Interaction	0.372	0.273	1.360	0.173	−0.163	0.908
	Treatment	−4.034	0.226	−17.830	0.000	−4.478	−3.590
	Time	−2.507	0.292	−8.570	0.000	−3.081	−1.933

PGR17	Interaction	3.442	2.722	1.260	0.206	−1.900	8.785
	Treatment	−5.307	2.164	−2.450	0.014	−9.555	−1.059
	Time	−15.652	2.854	−5.480	0.000	−21.255	−10.049

PGI	Interaction	0.251	1.073	0.230	0.815	−1.855	2.357
	Treatment	31.241	1.163	26.860	0.000	28.958	33.524
	Time	8.521	1.272	6.700	0.000	6.024	11.018

PGII	Interaction	0.843	1.154	0.730	0.465	−1.422	3.109
	Treatment	28.755	1.040	27.640	0.000	26.713	30.797
	Time	11.064	1.310	8.450	0.000	8.493	13.635

The article "Efficacy of Self-Made Hewei Decoction for Chronic Atrophic Gastritis and Its Effect on Gastrin and Pepsinogen Expression Levels" was retracted in 2023. Reasons: signs of a paper mill; suspected computer-generated content; unreliable results or conclusions; concerns about the data.

## Data Availability

The simulation experiment data used to support the findings of this study are available from the corresponding author upon request.
